The article "Effect of Combining Immersion Therapy with Shengji Ointment on Wound Healing Rate and Adverse Reaction Rate in Patients with Second-Degree Burn" was published in 2021. Journal: J Healthc Eng.

# Effect of Combining Immersion Therapy with Shengji Ointment on Wound Healing Rate and Adverse Reaction Rate in Patients with Second-Degree Burn

**DOI:** 10.1155/2021/1339683

**Published:** 2021-11-24

**Authors:** Yun Guo, Junjie Yu

**Affiliations:** Department of Burn, Affiliated Hospital of Jiangnan University, Wuxi 214122, Jiangsu Province, China

## Abstract

**Objective:**

To explore the effect of combining immersion therapy with Shengji ointment on wound healing rate and adverse reaction rate (ARR) in patients with second-degree burn.

**Methods:**

The data of 80 patients with second-degree burn treated in our hospital from February 2019 to February 2020 were retrospectively analyzed by the means of retrospective study, and the patients were equally divided into the treatment group and the control group according to their admission order, with 40 cases each. Immersion therapy was performed to all patients (7 d); after that, patients in the control group received routine medication (7 d), and those in the treatment group were treated with Shengji ointment until the wounds were healed, so as to compare their wound healing condition, ARRs, levels of inflammatory factors, and infection incidence.

**Results:**

Compared with the control group after treatment, the treatment group presented significantly shorter wound healing time (12.14 ± 1.26 vs. 15.98 ± 1.20, *P* < 0.001), better wound healing rate and quality (*P* < 0.05), and lower levels of inflammatory factors (*P* < 0.001); no significant between-group difference in ARRs was shown (*P* > 0.05); 34 patients in the treatment group (85.0%) and 26 patients in the control group (65.0%) had no infections, so the incidence rate of infections was significantly lower in the treatment group than in the control group (*P* < 0.05).

**Conclusion:**

Combining immersion therapy with Shengji ointment can reduce the levels of inflammatory factors in patients with second-degree burn, lower the incidence rate of infections, provide the conditions for wound healing, and increase the wound healing rate, which shall be promoted and applied in practice.

## 1. Introduction

Burn injury is tissue damage caused by heat, which is divided into first-degree burn, superficial second-degree burn, deep second-degree burn, and third-degree burn, of which the first-degree burn only injuries the epidermis and does not damage the germinal layer, so it can be healed in 3 to 5 days without scarring the skin [1, 2]. In the case of superficial and deep second-degree burns, patients' dermis and germinal layer are damaged, and epithelium regeneration can only rely on the residual germinal layer or appendages of skin; in the premise of timely treatment and no secondary infections, patients usually can be healed in 1–4 weeks [3, 4]. With poor treatment effect, wound surface infection or serious inflammatory reactions may occur and blood supply on wound surface will continue to deteriorate, causing necrosis of newborn tissue, arrest of epithelium growth, prolonged healing time, and even failure to natural healing and finally forming obvious scars [5]. Therefore, selecting suitable treatment modality and drugs to reduce the levels of inflammatory factors and prevent infections is the key to improving the wound healing rate in clinical treatment.

Wound healing belongs to the biological process in which multiple inflammatory factors and cytokines collectively participate, in which many inflammatory factors and cytokines are involved [6], so topical drugs are of great significance for wound recovery. The commonly used drug in current practice is silver sulfadiazine cream, which is able to absorb wound exudate and accelerate granulation proliferation, but it is easy to trigger infection and prolong the healing cycle; thus, the overall efficacy is unsatisfactory [7]. Scholars Fang M A et al used silver sulfadiazine as a control and applied the Qingre Shengji ointment that contained rhubarb, Chinese goldthread rhizome, baical skullcap root, and other herbs to rats with second-degree burn and found that the ointment could increase the content of vascular endothelial growth factor (VEGF) and hydroxyproline in wound and at the same time reduce the levels of interleukin-1 (IL-1) and tumor necrosis factor-*β* (TNF-*β*), thereby accelerating the wound healing for rats [8]. In addition, scholars Gravelier et al. also proved that Shaoshang Shengji ointment was able to effectively treat small area burns, cause less obvious scars, and present significant efficacy [9]. Previous studies have shown that application of Shengji ointment in patients with second-degree burns might be beneficial to improve their wound healing rate, but practice has indicated that the wound pain caused by burns can seriously affect the treatment willingness of patients, and some patients suffer from intolerable pain when changing fresh dressing, leading to poor treatment compliance [10, 11]. To improve the effect of topical drugs, some scholars suggested treating burn patients with immersion therapy and found that such therapy can easily remove the outer dressings, alleviate the pain from dressing changing, and completely clean the wound surface, which can effectively prevent infections.

In the review of previous literature, no studies have been found in academia combining the immersion therapy with Shengji ointment. Based on this, the actual effect of combining the two in wound healing of patients with second-degree burn was explored herein, with the results reported as follows.

## 2. Materials and Methods

### 2.1. Study Design

This retrospective study was conducted in our hospital from February 2019 to February 2020 to explore the effect of combining immersion therapy with Shengji ointment on wound healing rate and adverse reaction rate (ARR) in patients with second-degree burn. It was a double-blind study, meaning that neither the research objects nor researchers understood the trial grouping and the study designer was responsible for arranging and controlling the full trial.

### 2.2. Study Object Enrollment

The data of patients with second-degree burn treated in our hospital from February 2019 to February 2020 were retrospectively analyzed, and the patients were enrolled according to the following inclusion and exclusion criteria. Inclusion criteria: (1) the patients were diagnosed with second-degree burn after examination [11]; (2) the patients received treatment within 24 hours after injury and were treated in our hospital in the whole course without transferring to other hospitals during treatment or stopping treatment; (3) the patients did not present obvious shock; (4) the burn depth was relatively uniform, and the wound surface was red and white by observation; and (5) the patients were over 18 years old.

Exclusion criteria: (1) the patients could not communicate with others due to hearing disorders, language disorders, unconsciousness, mental diseases, or other factors; (2) the patients quit the trial in the middle of treatment due to ① progression disease during trial; ② severe complications; or ③ demand of quitting the trial; (3) the patients had severe organic diseases and other chronic underlying diseases that affect wound healing before burn; (4) the patients had severe inhalation injury; (5) the patients were using immunosuppresants; (6) the patients were pregnant or lactating women; and (7) the patients had severe malnutrition.

### 2.3. Steps

A total of 80 patients were enrolled in the study and equally divided into the trial group and the control group according to their treatment order, with 40 cases each. On the day that the patients agreed to join the study, the study team collected their sociodemographic data and clinical performance data, treated the patients by group, and measured their levels of inflammatory factors before and after treatment to calculate the incidence rates of infections and record the healing condition.

### 2.4. Moral Consideration

The study met the principles in *World Medical Association Declaration of Helsinki (2013)* [12]. After enrollment, the study team explained the study purpose, meaning, contents, and confidentiality to the patients and their family members and asked them to sign the informed consent.

### 2.5. Methods

All patients received the immersion therapy with the following steps: (1) completely disinfect the bathroom with chlorine-containing disinfectant (1 : 1,000), strictly implement the strategy of “one man, one bathtub” and keep the room temperature to about 30°C; (2) 30 min before immersion, intravenously infuse glucose saline to patients, then soak the affected part in mineral water, wait for 10 min until the patients adjust to it, and wipe up the dirt on body surface, internal dressing of wound, etc. In turns with sterile gloves, and change fresh mineral water to soak and wash the whole body; (3) measure the temperature of the patients; prepare the proper amount of normal saline according to their height, body mass, wound condition, etc., and mix with 0.5% povidone-iodine with the proportion of 9 : 1; then soak the affected part in it; and during the systemic therapy, keep the water temperature 1°C over the body temperature of patients to the greatest extent, and during the local therapy, 2°C, the patients could complained of the water temperature, and the maximum temperature should not be over 40°C; (4) during immersion, monitor the patients for vital sign changes and conduct caution catheter nursing for those with catheter indwelt; for patients with large area burn, prepare relevant first aid objects and glucose for their first immersion to prevent accident; (4) set the time for first immersion to be less than 20 min according to the patients' wound condition and tolerance; in the subsequent treatment, prolong the immersion time to 30 min as appropriate; (5) the patients received the immersion therapy for 7 consecutive days.

After 30 min of immersion, the compound bacteriolysis disinfectant was used to clean the wound surface by soaking, spaying, rinsing, and other methods to fully drain the secretion and clear away the necrotic tissue, and then the moisture on wound surface was absorbed with wet gauze. For the wounds with infection and suppuration, gentamicin injection (manufactured: Shandong Lukang Pharmaceutical Group, Saite Co., Ltd.; NMPA approval no. H37024046) could be applied to the wound surface and then wiped repeatedly with disinfection swab, and after washing, topical drugs could be applied. After cleaning, routine medication was conducted to patients in the control group, namely, applying 2% silver sulfadiazine cream (manufactured: Shandong Health Pharmaceutical Co., Ltd; NMPA approval no. H37020451) to the wound surface, binding up with sterile gauze, and keeping dressing change till 7 days after injury.

After immersion, the same cleaning method as the control group was conducted to patients in the treatment group, and then Shengji ointment therapy was performed with the following steps. (1) Shengji ointment contained rhubarb, Chinese goldthread rhizome, baical skullcap root, cape jasmine fruit, garden burnet root, lobular privet leaves (20 g each), 30 g of giant knotweed rhizome, 5 g of camphol, 1,000 ml of sesame oil, and proper amount of beeswax and white wax; the rhubarb, Chinese goldthread rhizome, baical skullcap root, cape jasmine fruit, garden burnet root, lobular privet leaves, and giant knotweed rhizome were soaked in the sesame oil, and camphol was ground into powder for standby application; after soaking for one week, the sesame oil containing the herbs was decocted on fire until the herbs were burnt, and then frankincense and myrrh were added and fired until they floated above the oil and then were filtered with gauze; finally, beeswax and white wax were added into the clean oil to extract the ointment. (2) After cleaning, the ointment was applied evenly to the affected part, and except for the beeswax and white wax, all herbs were ground to powder, disinfected with high pressure, and then sprayed on the wound surface. (3) If the wound was dry and scabbed, ointment change could be discontinued until the wound was healed; if the scabbed site was moist with excessive secretion, remove the scab and then apply the ointment and spray the powder until it was healed.

### 2.6. Observation Criteria

1. *General Information*. The general information extract form was established by the patients themselves, covering the inpatient number, name, gender, age, body mass, causes of burn, burn area, burn type, burn site, place of residence, and educational level.
2. *Wound Healing*. ① Wound healing time: the time from being injured to complete epithelization of wound; ② wound healing rate: mean wound healing rate = (wound area immediately after injury − wound area at each time phase)/wound area immediately after injury × 100%; ③ wound healing quality: the Vancouver scar scale (VSS) [13] was used as the basis for evaluating the color, thickness, vascularity, softness of the scar area after the wound was healed, and on a scale of 0–15 points, higher scores indicated more serious scars.
3. *ARR*. The adverse reactions occurred in patients of the two groups during treatment were recorded.
4. *Levels of Inflammatory Factors*. The patients' fasting venous blood in the morning was drawn before treatment (*T*_1_), 3 days after treatment (*T*_2_) and 7 days after treatment (*T*_3_) to measure their C-reactive protein (CRP) levels with immunoturbidimetry (kits manufactured by Nanjing Getein Biotech Inc., Jiangsu Changzhou MPA certification no. 20122400146) and TNF-*α*, IL-1, and IL-8 levels with chemiluminescence immunoassay (Cobase 411 analyzer with original supporting agents; NMPA (I) 20113402843).
5. *Incidence Rate of Infections*. The infections included marginal cellulitis, empyema under scab, newborn tissue necrosis, and others, and the numbers of patients with infections were counted.

### 2.7. Statistical Processing

In this study, the data processing software was SPSS20.0, the picture drawing software was GraphPad Prism 7 (GraphPad Software, San Diego, USA), the items included were enumeration data and measurement data, the methods used were *X*^2^ test and *t*-test, and differences were considered statistically significant at *P* < 0.05.

## 3. Results

### 3.1. General Information

The general information of patients in the two groups was not statistically different (*P* > 0.05) (see Table 1).

### 3.2. Comparison of Wound Healing

Compared with the control group, the treatment group presented significantly shorter wound healing time (*P* < 0.001) and better wound healing rate and quality (*P* < 0.05) (see Figure 1).

### 3.3. ARR

Patients in the two groups did not have serious adverse reactions. In the treatment group, 2 patients had erubescence (5.0%) and 1 patient had pruritus (2.5%); and in the control group, 4 patients had pruritus (10.0%). No significant between-group difference in ARR was presented (*P* > 0.05).

### 3.4. Comparison of Levels of Inflammatory Factors

After treatment, the levels of inflammatory factors were greatly lower in the treatment group than in the control group (*P* < 0.001) (see Figure 2).

### 3.5. Comparison of Incidence Rates of Infections

The incidence rates of infections were significantly lower in the treatment group than in the control group (*P* < 0.05) (see Figure 3).

In the treatment group, 2 patients had marginal cellulitis (5.0%), 1 patient had empyema under scab (2.5%), 2 patients had newborn tissue necrosis (5.0%), 1 patient had other infections (2.5%), and 34 patients had no infection (85.0%); and in the control group, 4 patients had marginal cellulitis (10.0%), 4 patients had empyema under scab (10.0%), 3 patients had newborn tissue necrosis (7.5%), 3 patients had other infections (7.5%), and 26 patients had no infection (65.0%).

## 4. Discussion

Burns are mostly caused by hot fluids, hot gases, etc., mild ones injure the skin and mucous membranes, and severe ones cause damage to the joints, muscles, and organs, which are relatively common tissue injury in the clinic. According to different burn degrees, the rule of three degrees and four levels is usually adopted internationally, which divides burns into the first-degree burn, superficial second-degree burn, deep second-degree burn, and third-degree burn [14], while on this basis, the Chinese Burn Association proposes the rule of five degrees and four levels [15], but the same definition of the second-degree burn remains the same, namely, superficial second-degree burn injures the superficial dermis and preserves some basal cells; and deep second-degree burn damages the deep dermis with some residual dermal reticular tissues. Because the dermis thickness is different in every part of the body, and the degree of burn caused by the same heat varies, the deep second-degree burn is prone to many variations, and the mild one is close to the superficial second-degree burn, while the severe one is close to the third-degree burn. Regardless of which, the germinal layer of patients with second-degree burn is damaged, and the superficial wounds with relatively less damage can heal spontaneously, but surgical treatment is required for the deep wounds, and postoperative frequent dressing changes are necessary to reduce the level of inflammatory factors. But from a practical point of view, most patients with second-degree burns tend to use wound medication alone, so it is the most dominant treatment modality in both surgical treatment and conservative treatment [16–18].

Second-degree burn wound usually remains hair follicles, sweat glands, and other tissues, so bacteria are extremely easy to breed, and some patients develop infections after pure medication on wounds, deepening the wound tissue gradually and slowing down the healing process. In addition, with the severe pain from dressing change, patients with second-degree burn have low compliance with wound medication, so the treatment effect of single wound medication is unsatisfactory. To improve their compliance, some scholars combined immersion therapy with wound medication due to the fact that immersion therapy can completely remove the wound pus, clean the necrotic tissue, improve the wound blood supply, and reduce the residual bacteria and toxin on the wound surface to prevent infection [19–21]. For patients who fear pain, proper thermal stimulation during immersion therapy can inhibit the excitement of cutaneous sensory nerve and interfere with nociceptive transmission and then alleviate the pain and enhance their compliance with dressing change [22]. It can be concluded from the study results herein that, after immersion therapy, the levels of inflammatory factors in patients of the two groups were reduced, indicating that such therapy had exact efficacy in alleviating inflammatory response. In addition, the levels were significantly lower in the treatment group than in the control group (*P* < 0.001), proving that the treatment effect of Shengji ointment was better than that of silver sulfadiazine cream.

Among the herbs contained in Shengji ointment, Chinese goldthread rhizome, baical skullcap root, and others can strongly inhibit *Pseudomonas aeruginosa*, Staphylococcus, and hemolytic Streptococcus and enhance the phagocytosis ability of reticuloendothelial system; rhubarb can hinder the generation of nucleic acid in bacterial cells and exert the antianaerobic effect; camphol can kill *Staphylococcus aureus* and ciridans streptococci; and it has been found by scholars Kim Eun Hee et al. that the antimicrobial spectrum of giant knotweed rhizome even contains resistant organism in hospital [23]. Combining multiple herbs effectively reduced the levels of inflammatory factors in patients and lowered the possibility of infections, and therefore the incidence rate of infections was greatly lower in the treatment group than in the control group (*P* < 0.05). Since wound healing is mainly divided into inflammatory reaction phase and proliferation repair phase, the reduction of inflammatory reaction can also improve the wound repair rate, and on the basis of the improvement of blood circulation in the patients' wound by immersion therapy, their tissue edema has been reduced, the drug absorption efficiency is higher, and with sesame oil promoting the granulation tissue growth of wound, the wound epithelialization has been accelerated, leading to shorter healing time. Not only that, sesame oil is also able to prolong the acid production of burn wounds, and acidified wounds can accelerate the release of oxyhemoglobin and benefit further healing, so the wound healing rate of the treatment group was significantly higher than that of the control group (*P* < 0.05).

In the study by scholars Ziwa et al., it was shown that Shengji ointment had the effect of healing and eschar separation [24], which was based on Suwen: Pibu Lun (plain questions: on cutaneous region). In this classic book, it was mentioned that invasion of pathogenic qi to skin leads to opening and dispersing of striae, opened and dispersed striae cause evils invading the vessels, and excess of pathogenic qi in vessels will then invade the channels. In TCM treatment, promoting blood circulation to remove blood stasis and eliminating evil and promoting granulation are also regarded as the substance, closely connecting the wound healing time with healing quality [25]. This study demonstrated that the treatment group presented remarkably higher wound healing quality than the control group (*P* < 0.001), demonstrating that Shengji ointment could improve wound healing for patients with higher safety and had exact clinical application value due to the fact that no obvious adverse reactions occurred in patients.

In conclusion, combining immersion therapy with Shengji ointment is conducive to improving wound healing for patients with second-degree burn, which shall be promoted and applied.

## Figures and Tables

**Figure 1:** Wound healing ($\bar{x}$ ±*s*). Note: # indicated P<0.05. (a) Wound healing time: the horizontal axis from left to right indicates the treatment group and the control group, and the vertical axis indicates time (d). The wound healing time was significantly lower in the treatment group than in the control group (12.14 ± 1.26 vs. 15.98 ± 1.20, *P* < 0.001). (b) Wound healing rate: the horizontal axis from left to right indicates the 3^rd^ day, 7^th^ day, and 14^th^ day, and the vertical axis indicates the rate (%); the black areas indicate the treatment group, and the gray areas indicate the control group. At the 3^rd^ day, 7^th^ day, and 14^th^ day, the wound healing rates were significantly higher in the treatment group than in the control group (28.12 ± 2.14 vs. 20.15 ± 2.35, 56.98 ± 5.57 vs. 41.58 ± 4.68, 85.23 ± 5.47 vs. 78.98 ± 4.50, *P* < 0.05). (c) Wound healing quality: the horizontal axis from left to right indicates the color, thickness, vascularity, and softness, and the vertical axis indicates the VSS (points); the black areas indicate the treatment group, and the gray areas indicate the control group. The scores on color, thickness, vascularity, and softness were obviously higher in the treatment group than in the control group (2.07 ± 0.24 vs. 3.08 ± 0.35, 1.35 ± 0.25 vs. 1.69 ± 0.35, 1.23 ± 0.21 vs. 1.52 ± 0.35, 2.34 ± 0.20 vs. 2.70 ± 0.48, *P* < 0.001).

**Figure 2:** Comparison of levels of inflammatory factors ($\bar{x}$±*s*, *μ*g/L). (a–d) The horizontal axes from left to right indicated *T*_1_, *T*_2_, and *T*_3_, and the vertical axes indicated the levels of inflammatory factors; the lines with dots indicated the treatment group, and the lines with blocks indicated the control group; and # indicated *P* < 0.001. (a) CRP levels. At *T*_1_, no statistical difference in CRP levels between the treatment group and the control group was presented (7.90 ± 0.45 vs. 7.92 ± 0.41, *P* > 0.05); and at *T*_2_ and *T*_3_, the CRP levels were greatly lower in the treatment group than in the control group (4.26 ± 0.34 vs. 5.68 ± 0.47 and 2.24 ± 0.24 vs. 3.57 ± 0.35, *P* < 0.001). (b) TNF-*α* levels. At *T*_1_, no statistical difference in TNF-*α* levels between the treatment group and the control group was presented (65.12 ± 5.98 vs. 65.20 ± 5.14, *P* > 0.05); and at *T*_2_ and *T*_3_, the TNF-*α* levels were greatly lower in the treatment group than in the control group (35.65 ± 4.20 vs. 56.75 ± 4.98 and 28.98 ± 2.68 vs. 38.98 ± 4.68, *P* < 0.001). (c) IL-1 levels. At *T*_1_, no statistical difference in IL-1 levels between the treatment group and the control group was presented (130.58 ± 10.65 vs. 130.53 ± 10.47, *P* > 0.05), and at *T*_2_ and *T*_3_, the IL-1 levels were greatly lower in the treatment group than in the control group (64.98 ± 5.10 vs. 80.66 ± 7.65 and 35.56 ± 3.65 vs. 46.98 ± 5.40, *P* < 0.001). (d) IL-8 levels. At *T*_1_, no statistical difference in IL-8 levels between the treatment group and the control group was presented (120.98 ± 10.35 vs. 120.86 ± 10.24, *P* > 0.05), and at *T*_2_ and *T*_3_, the IL-8 levels were greatly lower in the treatment group than in the control group (65.98 ± 8.96 vs. 86.21 ± 11.65 and 36.98 ± 3.21 vs. 51.98 ± 4.68, *P* < 0.001).

**Figure 3:** Comparison of incidence rates of infections (n(%)). The black areas indicate marginal cellulitis, the dark gray areas indicate empyema under scab, the white areas indicate newborn tissue necrosis, the grid areas indicate other infections, and the light gray areas indicate no infection; the left figure indicated the treatment group, and the right figure indicated the control group.

**Table 1:** General information.

Group	Treatment (*n* = 40)	Control (*n* = 40)	*X* ^2^/*t*	*P*
Gender			0.061	0.805
Male	28	29		
Female	12	11		
Age (years)				
Range	18–48	19–50		
Mean age	34.58 ± 1.68	34.64 ± 1.75	0.118	0.906
Mean body mass (kg)	62.98 ± 2.12	62.95 ± 2.10	0.064	0.950
Cause of burn				
Flame	20	22	0.201	0.654
Hot liquid	12	13	0.058	0.809
Electric arc	5	4	0.125	0.723
Chemical	3	1	1.053	0.305
Burn area (%)	24.24 ± 2.68	24.30 ± 2.74	0.099	0.921
Burn type			0.201	0.654
Deep second-degree burn	20	18		
Superficial second-degree burn	20	22		
Burn part				
Upper/lower limb	24	26	0.213	0.644
Head and face	10	10	0.000	1.000
Trunk	6	4	0.457	0.499
Place of residence			0.058	0.809
Urban area	28	27		
Rural area	12	13		
Educational level				
Senior high school and below	15	18	0.464	0.496
Junior college	16	15	0.053	0.818
College and above	9	7	0.313	0.576

## Data Availability

The data used to support the findings of this study are available from the corresponding author upon request.
